# Identification of Molecular Biomarkers and Key Pathways for Esophageal Carcinoma (EsC): A Bioinformatics Approach

**DOI:** 10.1155/2022/5908402

**Published:** 2022-01-12

**Authors:** Md. Rakibul Islam, Mohammad Khursheed Alam, Bikash Kumar Paul, Deepika Koundal, Atef Zaguia, Kawsar Ahmed

**Affiliations:** ^1^Department of Software Engineering, Daffodil International University (DIU), Ashulia, Savar, Dhaka 1342, Bangladesh; ^2^Preventive Dentistry Department, College of Dentistry, Jouf University, Sakaka 72345, Saudi Arabia; ^3^Center for Transdisciplinary Research (CFTR), Saveetha Dental College, Saveetha Institute of Medical and Technical Sciences, Saveetha University, Chennai, India; ^4^Department of Public Health, Faculty of Allied Health Sciences, Daffodil International University, Dhaka, Bangladesh; ^5^Group of Bio-Photomatix, Department of Information and Communication Technology, Mawlana Bhashani Science and Technology University, Santosh, Tangail 1902, Bangladesh; ^6^Department of Systemics, School of Computer Science, University of Petroleum and Energy Studies, Dehradun, Uttarakhand 248007, India; ^7^Department of Computer Science, College of Computers and Information Technology, Taif University, P.O. Box 11099, Taif 21944, Saudi Arabia; ^8^Department of Electrical and Computer Engineering, University of Saskatchewan, 57 Campus Drive, Saskatoon, SK, Canada S7N 5A9

## Abstract

Esophageal carcinoma (EsC) is a member of the cancer group that occurs in the esophagus; globally, it is known as one of the fatal malignancies. In this study, we used gene expression analysis to identify molecular biomarkers to propose therapeutic targets for the development of novel drugs. We consider EsC associated four different microarray datasets from the gene expression omnibus database. Statistical analysis is performed using R language and identified a total of 1083 differentially expressed genes (DEGs) in which 380 are overexpressed and 703 are underexpressed. The functional study is performed with the identified DEGs to screen significant Gene Ontology (GO) terms and associated pathways using the Database for Annotation, Visualization, and Integrated Discovery repository (DAVID). The analysis revealed that the overexpressed DEGs are principally connected with the protein export, axon guidance pathway, and the downexpressed DEGs are principally connected with the L13a-mediated translational silencing of ceruloplasmin expression, formation of a pool of free 40S subunits pathway. The STRING database used to collect protein-protein interaction (PPI) network information and visualize it with the Cytoscape software. We found 10 hub genes from the PPI network considering three methods in which the interleukin 6 (IL6) gene is the top in all methods. From the PPI, we found that identified clusters are associated with the complex I biogenesis, ubiquitination and proteasome degradation, signaling by interleukins, and Notch-HLH transcription pathway. The identified biomarkers and pathways may play an important role in the future for developing drugs for the EsC.

## 1. Introduction

Esophageal carcinoma (EsC) is a member of the cancer group that occurs in the esophagus; globally, it is known as one of the fatal malignancies. In the year of 2018, EsC ranked as the ninth most common type of cancer with 572,000 new cases (3.72% of all types of cancer cases) and the sixth most common form of cancer in mortality with 509,000 deaths [1]. EsC remains an endemic disease in several parts of the world especially in third world countries [2]. Though the incidence rates of EsC are unstable worldwide with the highest rates of incidence were found in Africa and eastern Asia [1]. Gender-wise studies claimed that around 70% of EsC patients are male [1]. Drinking alcohol and smoking are listed as risk factors for esophageal squamous cell carcinoma in the United States [3]. Gastroesophageal reflux disease (GERD) and Barrett's esophagus are connected with an increased risk of the development of EsC [4, 5]. Obesity also accounts as a risk factor of esophagus-related adenocarcinoma [6]. EsC remains a global concern for its lower survival rate, 5-year survival rates until now stayed less than 20% [7]. Though a huge improvement had occurred in the medical field over the last few decades, the median survival rates of EsC have been slightly grown in the last few years [8]. Most of the EsC cases are diagnosed in its latter stages for the lack of early clinical symptoms. Some common symptoms are accounted such as sudden weight loss, breastbone burn feel, chest pain, and dysphagia. Microarray gene expression profile and gene chip analysis have been hugely applied in the medical field [9]. Gene expression analysis helps to decode differentially expressed genes and molecular biomarkers using several techniques that may have a potential influence on cancer development [10]. Molecular biomarkers acted a significant role with an early diagnostic and prognostic value in cancer treatment. A few studies have been produced to identify molecular biomarkers for EsC. In a study, Dong et al. showed that Methyltransferase Like 7B can take part in the early detection of esophageal adenocarcinoma [11]. Wang et al. claimed that the MAPK1 gene showed abnormal expression which may contribute to the development of EsC [12]. EsC is one of the cancers that take lots of attention from the researchers but still not much known about its mechanism and progression. The increasing study of EsC-associated molecular biomarkers may provide a foundation for unique approaches in preventing, diagnosing, and treating EsC. In this study, we have conducted a comprehensive microarray-based genome-wide analysis to identify molecular signatures using bioinformatics methods and tools. The current study is started by collecting 4 EsC-associated microarray datasets. We identified differentially expressed genes (DEGs) from datasets. DEGs are presented to complete functional study and protein-protein interaction analysis. Significant clusters are identified from protein interaction networks. We also identified hub genes using connectivity value, maximum neighborhood component (MNC), and bottleneck methods.

## 2. Methodology

### 2.1. Microarray Data Collection

Many studies have been conducted on esophageal cancer to explore genetic biomarkers [13–15]. But there are very few numbers of comprehensive analyses on EsC so that the exact genetic mechanisms are remained unknown till now. To explore genetic biomarkers, we applied a comprehensive analysis in our current study. We used four different microarray datasets to complete this study. GSE93756, GSE94012, GSE104958, and GSE143822 datasets are selected from National Center for Biotechnology Information's (NCBI) Gene Expression Omnibus (GEO, https://www.ncbi.nlm.nih.gov/geo/) [16]. GSE93756 dataset has four samples based on platform GPL21282 Phalanx Human OneArray Ver. 7 Release 1. GSE94012 dataset has six samples based on platform GPL15207 [PrimeView] Affymetrix Human Gene Expression Array. GSE104958 dataset has a total of 46 samples, and the dataset is based on platform GPL21185 Agilent-072363 SurePrint G3 Human GE v3 8x60K Microarray 039494 (Probe Name Version) [17]. GSE143822 dataset has eight samples, and it is based on platform GPL20844 Agilent-072363 SurePrint G3 Human GE v3 8x60K Microarray 039494. Step by step process of this study is demonstrated in Figure 1.

### 2.2. Data Processing and DEG Identification

Limma stands for linear models for microarray data, and most of the functionality of limma has been developed for microarray data. Using limma for microarray data processing is simple, and its result is mostly accurate. We used the limma package of the R language to convert the raw files of our selected four datasets [18]. The datasets are converted into gene expression measures for further analysis. To identify statistical significance of genes log 2 FC (fold change) > 1.50 for overexpression, log 2 FC < −1.50 for downexpression, and standard adjusted *P* value < 0.05 are applied [19, 20].

### 2.3. GO and Pathway Enrichment Analysis of DEGs

Gene Ontology (GO) analysis provides wide biological exploration outcomes for a single gene or gene set. In recent years, GO analysis is a crucial part of system biology-related studies. In another corner, pathway enrichment analysis assists in explore mechanistically insight between gene sets produced from the wide genome-scale analysis [21]. In this study, we used the Gene Ontology database to explore DEGs associated GO terms [22], and pathway analysis is conducted using Kyoto Encyclopedia of Genes and Genomes (KEGG) [23], REACTOME [24], BIOCARTA [25], and Biological Biochemical Image Database (BBID) [26] databases. The Database for Annotation, Visualization, and Integrated Discovery (DAVID, http://david.abcc.ncifcrf.gov/) is fruitful to gather all outcomes [27]. Statistical significance *P* value < 0.05 is maintained for identifying the final outcomes.

### 2.4. PPI Construction and Clustering Analysis

The Search Tool for the Retrieval of Interacting Genes/Proteins (STRING, https://string-db.org/) repository is used to explore internal interactions between DEGs [28]. A high combine score > 0.70 is used to validate the interactions. Open-source software Cytoscape [29] is used to generate the protein-protein interaction (PPI) networks. CytoHubba plugin is applied to get topological parameter value [30]. To identify clusters from PPI networks, we used the Molecular Complex Detection (MCODE) algorithm [31]. The MCODE plugin built-in parameter is used for the analysis degree cutoff = 2, node score cutoff = 0.2, *k* − core = 2, and maximum depth = 100 is counted as a minimum criterion. The functional pathway analysis in the cluster is performed by using the REACTOME database.

## 3. Result and Demonstration

### 3.1. DEG Screening

Initially, a total of 20102, 20085, 33762, and 32212 DEGs are identified from GSE93756, GSE94012, GSE104958, and GSE143822 datasets. After applying the minimum log (FC) and *P* value criterion, 5802, 5393, 5945, and 7024 DEGs are identified correspondingly. 380 upregulated and 703 downregulated DEGs are screened out in selected four datasets that are used for further analysis (Table 1). The top 10 upregulated and downregulated DEGs are shown in Table 2.

### 3.2. GO and Pathway Enrichment Analysis of DEGs

We applied functional analysis using the DAVID database to achieve further knowledge into the function of identified DEGs. The functional analysis reveals significant enriched GO terms and pathways of identified DEGs. The GO analysis explores that the overexpressed DEGs are mainly associated with protein ubiquitination, and regulation of cell cycle for biological process (BP); endoplasmic reticulum membrane and nucleoplasm for cellular component (CC); and protein binding, DNA binding for molecular function (MF) (Table 3, Figure 2). On another chapter of GO analysis explores the downexpressed DEGs associated with the translational initiation and SRP-dependent cotranslational protein targeting to membrane for BP; extracellular matrix, and ribosome for CC; structural constituent of ribosome, and NADH dehydrogenase (ubiquinone) activity for MF (Table 4, Figure 3).

We used four different databases to achieve the associated pathways more clearly. The pathway analysis revealed that the overexpressed DEGs are principally connected with the protein export, axon guidance, and RHO GTPases Activate Formins pathway (Table 5(a), Figure 4); the downexpressed DEGs are principally connected with the L13a-mediated translational silencing of ceruloplasmin expression, formation of a pool of free 40S subunits, and GTP hydrolysis and joining of the 60S ribosomal subunit pathways (Table 5(b), Figure 5).

### 3.3. PPI Construction and Hub Gene Identifications

Using the STRING database, we generated the PPI network and visualized with Cytoscape software. Constructed PPI network has 646 nodes and 2055 connections, including 172 upregulated DEGs and 474 downregulated DEGs (Figure 6). Using CytoHubba plugin, we identified the top 10 hub genes from the PPI network including IL6, CDH1, NOTCH1, ATP5C1, BPTF, MRPS11, MRPS15, MRPL1, NDUFB7, and NDUFS5. CytoHubba plugin has 11 different methods to identify significant genes from the PPI network; in this study, we consider three methods including connectivity value (degree), maximum neighborhood component (MNC), and bottleneck to identify hub genes. In the PPI network, the IL6 gene has the highest number of degree value 68, MNC value 60, and bottleneck value 151 (Figure 7). The top 10 hub gene name and their rank based on three methods are screened in Table 6.

### 3.4. Clustering Analysis

Cluster analysis is conducted using the MCODE method. In this analysis, 11 clusters are identified where the number of nodes is greater than 5. We identified four significant clusters from the constructed PPI network. The most significant cluster is enriched with MCODE score 17.5 and node density 33; 2nd significant cluster has MCODE score 12 and node density 12; 3rd significant cluster has MCODE score 9.238 and node density 22; the 4th significant cluster has MCODE score 5 and node density 9. Pathway enrichment analysis explored that clusters are significantly enriched with the complex I biogenesis, mitochondrial translation termination, ubiquitination and proteasome degradation, signaling by interleukins, and Notch-HLH transcription pathway (Table 7). Cluster outcomes with their associated pathways are shown in Figure 8.

## 4. Discussion

Globally EsC is considered one of the most deadly diseases for its fast development and base presage. Around 80% of EsC cases are recorded from less developed regions in the world [2]. In 2012 in China, EsC had listed the fifth common diagnosed cancer type and the fourth eminent cause of mortality [32]. It is urgent to understand the clinical epidemiology of EsC to develop medical treatment. In this study, we developed a microarray gene profile analysis to identify molecular signatures. EsC-associated four different datasets GSE93756, GSE94012, GSE104958, and GSE143822 are selected, and these datasets are analyzed with the limma package of R language. 380 upregulated and 703 downregulated DEGs are matched in all datasets following every criterion. These DEGs are applied to draw significant GO terms using the DAVID database. GO analysis shows that the upregulated DEGs are associated with protein ubiquitination, regulation of cell cycle, endoplasmic reticulum membrane, nucleoplasm, and protein binding. The downregulated DEGs are associated with translational initiation, SRP-dependent cotranslational protein targeting to membrane, extracellular matrix, ribosome, and structural constituent of ribosome. Cell cycle abnormalities had been indicated as a key factor of esophagus tumorigenesis [33, 34]. In 2017, Otto et al. claimed that the cell cycle protein may play a promising role in cancer therapy [35].

In this study, PPI network is constructed by using identified DEGs. From the PPI network, we found 10 hub genes (IL6, CDH1, NOTCH1, ATP5C1, BPTF, MRPS11, MRPS15, MRPL1, NDUFB7, and NDUFS5) using three combined methods. Interleukin 6 (IL6) gene is a member of the Interleukin family, and it takes part in cell growth operation. IL6 can act as both a proinflammatory cytokine and an anti-inflammatory myokine, and it is associated with many types of cancer development [36]. A study showed that breast cancer cells produced IL6 as a core compound [37]. IL6 also listed as a therapeutic biomarker in renal cell carcinoma [38]. IL6 shows poor prognosis values in lung cancer patients [39]. IL6-associated signaling pathways also take part in cancer progression. Based on the above discussion, we can say that IL6 may play a significant role in EsC progression. Cadherin 1 (CDH1) gene is connected with protein-coding. CDH1 is associated with the cell proliferation pathway, which plays an important preface in cancer development [40]. Mutations of CDH1 protein marked as an increased risk factor for hereditary diffuse gastric cancer (HDRC) [41, 42].

HDRC affected women to embrace a high risk of having breast cancer [43]. HDRC patients increased high risk of developing stomach cancer which is associated with the esophagus organ. Several characteristics indicate that CDH1 may take part in the development of EsC. NOTCH1 is known for encoding the NOTCH family of proteins. NOTCH1 plays a role in cell growth and proliferation, differentiation, and apoptosis. NOTCH1 is engaged in many types of cancer, including triple-negative breast cancer, leukemia, brain tumors, and many others. It influences apoptosis, proliferation, immune response, and the population of cancer stem cells [44]. Regarding the above discussion, we can assume NOTCH1 may impact EsC development. The Bromodomain PHD Finger Transcription Factor (BPTF) gene was found overexpressed and showed poor prognosis value in the tissue of lung adenocarcinoma [45]. A study from 2015 proposed BPTF as a novel target for anticancer therapy [46].

In the PPI analysis section, we applied the MCODE method to identify clusters. Significant four clusters are identified, and pathway analysis is performed. Pathway analysis showed that the clusters are principally enriched with complex I biogenesis, mitochondrial translation termination, mitochondrial translation initiation, and interferon-alpha/beta signaling pathway. Mitochondrial biogenesis develops breast cancer tumors in the epithelial cell lines [47].

The authors believe the outcomes of this study will make an impact on the biomarker identification of EsC. But more studies are required to prove the statement. Lack of tools and established laboratory, we could not verify our outcomes which is the limitation of this study. For future goals, we will use the outputs to explore microRNA biomarkers for EsC, which will give us deeper knowledge regarding EsC development.

## Figures and Tables

**Figure 1:** Flow diagram of this study. This diagram explains we start our first step of this study from the GEO database; from the database, we select 4 datasets for statistical analysis and identify DEGs maintaining our cut-off filtration. After that, we categorize the identified DEGs according to their expression (upregulated and downregulated). After categorization, we implement function analysis and protein-protein interaction analysis, which are the two most key analyses of this study.

**Figure 2:** Gene Ontology analysis of upregulated DEGs using DAVID functional tools. Different colors of dots mean different categories of GO terms. The green-colored dot indicates biological process, the blue-colored dot indicates cellular component, and the red-colored dot defines molecular functions. The *x*-axis indicates the |Log (*P* value)| of associated GO terms. *y*-axis indicates the GO term name. The size of a dot represents gene count.

**Figure 3:** Gene Ontology analysis of downregulated DEGs using DAVID functional tools. Different colors of dots mean different categories of GO terms. The green-colored dot indicates biological process, the blue-colored dot indicates cellular component, and the red-colored dot defines molecular functions. The *x*-axis indicates the |Log (*P* value)| of associated GO terms. *y*-axis indicates the GO term name. The size of a dot represents gene count.

**Figure 4:** Bar plot diagram to demonstrate pathway analysis outcomes of upregulated DEGs. Different color of bars indicates the different database name. The *x*-axis indicates the value of |log10 (*P* value)|, and *y*-axis indicates the pathway term name.

**Figure 5:** Bar plot diagram to demonstrate pathway analysis outcomes of downregulated DEGs. Different color of bars indicates the different database name. The *x*-axis indicates the value of |log10 (*P* value)|, and *y*-axis indicates the pathway term name.

**Figure 6:** PPI network using identified DEGs. Nodes represent DEGs, and edge represents the connection between DEGs. The network has 646 nodes and 2055 connections. Green nodes represent upregulated DEGs, and red nodes represent downregulated DEGs. Eclipse-shaped nodes indicate the hub genes of the network. Hub genes are explored using 3 combined methods.

**Figure 7:** Bar plot diagram to represent the values of degree, MNC, and bottleneck for specific hub genes. The red bar indicates degree value, the blue bar indicates MNC value, and the black bar indicates bottleneck value. The *x*-axis represents the gene name, and the *y*-axis represents numerical values of the corresponding method.

**Figure 8:** Top 4 clusters and their associated pathways for (a) cluster 1, (b) cluster 2, (c) cluster 3, and (d) cluster 4. Hexagonal-shaped nodes present pathway name, and eclipse-shaped presents the gene name.

**Table 1:** Dataset analysis details (a) before filtration and (b) after filtration.

Accession number	Amount of sample	Upregulated DEGs	Downregulated DEGs	Total DEGs
(A) Before logFC filtration				
GSE93756	4 samples	6197	13905	20102
GSE94012	6 samples	4464	15621	20085
GSE104958	46 samples	22238	11524	33762
GSE143822	8 samples	14552	17660	32212
Overlapped		1003	3818	4821
(B) After logFC filtration				
GSE93756	4 samples	1094	4708	5802
GSE94012	6 samples	1520	3873	5393
GSE104958	46 samples	1128	4617	5945
GSE143822	8 samples	841	6183	7024
Overlapped		380	703	1083

**Table 2:** Top 10 (a) upregulated and (b) downregulated DEG name and LogFC value.

DEG symbol	LogFC
(A) Upregulated DEGs	
AFG3L2	8.456189
CAMKK2	8.268455
EIF4H	6.039133
SLC6A19	5.983653
OR2L3	5.71944
FUNDC2P2	5.401373
KRT6B	5.195899
WRAP53	5.106136
OR56A3	5.054809
LINC01465	5.031665
(B) Downregulated DEGs	
COPS5	-11.2045
C3orf59	-9.20752
NOX6	-8.2488
RAB3B	-7.23927
LINC01279	-6.98733
NEDD5	-6.46107
USP26	-6.41274
TTLL9	-6.22158
NKD1	-6.09627
FCAR	-6.01488

**Table 3:** Gene Ontology analysis of upregulated DEGs using DAVID functional tools.

Category	GO ID	GO term	Count	%	*P* value
BP	GO:0045892	Negative regulation of transcription, DNA-templated	22	0.035989	0.001478
BP	GO:0046513	Ceramide biosynthetic process	5	0.008179	0.001541
BP	GO:0016567	Protein ubiquitination	17	0.02781	0.00305
BP	GO:0051726	Regulation of cell cycle	9	0.014723	0.003954
BP	GO:0048013	Ephrin receptor signaling pathway	7	0.011451	0.008317
BP	GO:0016477	Cell migration	10	0.016359	0.008953
BP	GO:0000045	Autophagosome assembly	5	0.008179	0.009555
BP	GO:0045893	Positive regulation of transcription, DNA-templated	20	0.032717	0.009702
BP	GO:0055007	Cardiac muscle cell differentiation	4	0.006543	0.017191
BP	GO:0051865	Protein autoubiquitination	5	0.008179	0.018845
CC	GO:0005789	Endoplasmic reticulum membrane	37	0.060527	1.84E-05
CC	GO:0005654	Nucleoplasm	83	0.135776	8.75E-05
CC	GO:0005634	Nucleus	136	0.222477	7.26E-04
CC	GO:0005802	Trans-Golgi network	10	0.016359	0.001509
CC	GO:0031965	Nuclear membrane	13	0.021266	0.002026
CC	GO:0005622	Intracellular	39	0.063798	0.013664
CC	GO:0005737	Cytoplasm	123	0.201211	0.015049
CC	GO:0005829	Cytosol	80	0.130869	0.036397
CC	GO:0005671	Ada2/Gcn5/Ada3 transcription activator complex	3	0.004908	0.038709
CC	GO:0000139	Golgi membrane	19	0.031081	0.046953
MF	GO:0005515	Protein binding	237	0.387698	1.25E-08
MF	GO:0003677	DNA binding	56	0.091608	5.22E-04
MF	GO:0003684	Damaged DNA binding	7	0.011451	0.002026
MF	GO:0004842	Ubiquitin-protein transferase activity	16	0.026174	0.004151
MF	GO:0061630	Ubiquitin protein ligase activity	11	0.017994	0.00625
MF	GO:0005070	SH3/SH2 adaptor activity	6	0.009815	0.006276
MF	GO:0008565	Protein transporter activity	6	0.009815	0.017551
MF	GO:0017137	Rab GTPase binding	8	0.013087	0.022939
MF	GO:0003676	Nucleic acid binding	31	0.050712	0.02606
MF	GO:0032794	GTPase activating protein binding	3	0.004908	0.03379

∗GO: Gene Ontology; ∗BP: biological process; ∗CC: cellular component; ∗MF: molecular function.

**Table 4:** Gene Ontology analysis of downregulated DEGs using DAVID functional tools.

Category	GO ID	Term	Count	%	*P* value
BP	GO:0006413	Translational initiation	37	0.014347	4.26E-09
BP	GO:0006614	SRP-dependent cotranslational protein targeting to membrane	27	0.010469	1.96E-07
BP	GO:0006412	Translation	50	0.019388	3.60E-07
BP	GO:0019083	Viral transcription	29	0.011245	6.66E-07
BP	GO:0000184	Nuclear-transcribed mRNA catabolic process, nonsense-mediated decay	30	0.011633	7.51E-07
BP	GO:0048245	Eosinophil chemotaxis	8	0.003102	1.64E-06
BP	GO:0007155	Cell adhesion	69	0.026755	4.88E-05
BP	GO:0006364	rRNA processing	38	0.014735	1.20E-04
BP	GO:0002548	Monocyte chemotaxis	13	0.005041	2.75E-04
BP	GO:0007156	Homophilic cell adhesion via plasma membrane adhesion molecules	29	0.011245	5.11E-04
Category		Term	Count	%	*P* value
CC	GO:0031012	Extracellular matrix	55	0.021326	3.51E-07
CC	GO:0005840	Ribosome	37	0.014347	4.78E-07
CC	GO:0022625	Cytosolic large ribosomal subunit	20	0.007755	5.24E-06
CC	GO:0030424	Axon	40	0.01551	3.48E-05
CC	GO:0005578	Proteinaceous extracellular matrix	45	0.017449	6.17E-05
CC	GO:0005788	Endoplasmic reticulum lumen	35	0.013571	9.14E-05
CC	GO:0005747	Mitochondrial respiratory chain complex I	14	0.005429	2.80E-04
CC	GO:0022627	Cytosolic small ribosomal subunit	13	0.005041	8.53E-04
CC	GO:0098793	Presynapse	15	0.005816	0.001358
CC	GO:0015935	Small ribosomal subunit	9	0.00349	0.00193
Category		Term	Count	%	*P* value
MF	GO:0003735	Structural constituent of ribosome	49	0.019	1.85E-08
MF	GO:0008137	NADH dehydrogenase (ubiquinone) activity	13	0.005041	0.001124
MF	GO:0044822	Poly(A) RNA binding	134	0.051959	0.001979
MF	GO:0008237	Metallopeptidase activity	17	0.006592	0.002751
MF	GO:0005201	Extracellular matrix structural constituent	15	0.005816	0.002881
MF	GO:0003723	RNA binding	70	0.027143	0.004922
MF	GO:0047555	3′,5′-cyclic-GMP phosphodiesterase activity	6	0.002327	0.006619
MF	GO:0042056	Chemoattractant activity	8	0.003102	0.009717
MF	GO:0001077	Transcriptional activator activity, RNA polymerase II core promoter proximal region sequence-specific binding	34	0.013184	0.01087
MF	GO:0008009	Chemokine activity	11	0.004265	0.012935

**Table 5:** Pathway enrichment analysis of (a) upregulated and (b) downregulated DEGs using DAVID functional tools.

Pathway term	Benjamini	*P* value	Source
(A) Upregulated			
Protein export	0.169923	9.40E-04	KEGG
Axon guidance	0.284819	0.00338	KEGG
RHO GTPases Activate Formins	0.959243	0.007813	REACTOME
HATs acetylate histones	0.882682	0.010449	REACTOME
Sphingolipid metabolism	0.583473	0.013182	KEGG
Pathogenic Escherichia coli infection	0.580496	0.017396	KEGG
Golgi associated vesicle biogenesis	0.975818	0.026998	REACTOME
ErbB signaling pathway	0.671562	0.027725	KEGG
Sphingolipid signaling pathway	0.637004	0.030241	KEGG
XBP1(S) activates chaperone genes	0.956916	0.030359	REACTOME
Lysosome	0.593513	0.031324	KEGG
The information-processing pathway at the IFN-beta enhancer	0.978374	0.034876	BIOCARTA
Activation of RAC1	0.961151	0.039023	REACTOME
Signaling of hepatocyte growth factor receptor	0.890962	0.040208	BIOCARTA
Epithelial cell signaling in helicobacter pylori infection	0.654812	0.042066	KEGG
(B) Downregulated			
L13a-mediated translational silencing of ceruloplasmin expression	3.71E-07	4.17E-10	REACTOME
Formation of a pool of free 40S subunits	4.51E-07	5.06E-10	REACTOME
GTP hydrolysis and joining of the 60S ribosomal subunit	4.84E-07	5.43E-10	REACTOME
Ribosome	3.48E-07	1.26E-09	KEGG
Peptide chain elongation	4.55E-06	5.11E-09	REACTOME
Selenocysteine synthesis	1.04E-05	1.17E-08	REACTOME
Eukaryotic translation termination	1.37E-05	1.53E-08	REACTOME
Viral mRNA translation	1.99E-05	2.24E-08	REACTOME
Nonsense mediated decay (NMD) independent of the exon junction complex (EJC)	2.30E-05	2.58E-08	REACTOME
SRP-dependent cotranslational protein targeting to membrane	3.08E-04	3.45E-07	REACTOME
Nonsense mediated decay (NMD) enhanced by the exon junction complex (EJC)	3.78E-04	4.24E-07	REACTOME
Formation of the ternary complex, and subsequently, the 43S complex	0.008265	9.31E-06	REACTOME
Ribosomal scanning and start codon recognition	0.012429	1.40E-05	REACTOME
Translation initiation complex formation	0.012429	1.40E-05	REACTOME
Chemokine	0.001886	3.85E-05	BBID

**Table 6:** Rank of 10 hub genes based on degree, MNC, and bottleneck methods.

Gene name	Rank degree	Rank MNC	Rank bottleneck
IL6	1	1	1
CDH1	2	3	2
NOTCH1	3	2	3
ATP5C1	4	4	5
BPTF	5	10	4
MRPS11	6	5	6
MRPS15	7	6	8
MRPL1	8	7	9
NDUFB7	9	8	7
NDUFS5	10	9	10

**Table 7:** Associated pathways of significant 4 clusters.

Pathway terms	Count	%	*P* value
(A) Cluster 1			
Complex I biogenesis	15	45.45455	6.48E-24
Mitochondrial translation termination	15	45.45455	6.35E-21
Mitochondrial translation initiation	15	45.45455	6.35E-21
Mitochondrial translation elongation	15	45.45455	6.35E-21
Respiratory electron transport	13	39.39394	3.91E-17
(B) Cluster 2			
Ubiquitination and proteasome degradation	12	0.593178	5.78E-17
(C) Cluster 3			
Interferon alpha/beta signaling	9	0.3159	1.32E-13
Signaling by interleukins	3	0.1053	0.003542
ISG15 antiviral mechanism	3	0.1053	0.008028
(D) Cluster 4			
B-WICH complex positively regulates rRNA expression	3	0.194805	9.95E-05
Notch-HLH transcription pathway	2	0.12987	0.002863

## Data Availability

The datasets used and/or analyzed during the current study are available from the corresponding author on reasonable request.
